# Influence of Internet Language Violence on Young Students' Mental Health and Intervention Countermeasures

This article has been retracted.

**DOI:** 10.1155/2021/1603117

**Published:** 2021-11-10

**Authors:** Xiaoqin Shi, Chao Yu, Dongmei Wu

**Affiliations:** ^1^College of Languages and Culture, Northwest A&F University, Yangling 712100, Shaanxi, China; ^2^College of Psychology, Yichun University, Yichun 333600, Jiangxi, China; ^3^College of Education, Minzu University of China, Peking 100081, China

## Abstract

With the development of the Internet, it has increasingly become an indispensable product in people's lives, but many problems have arisen with it. Internet language violence is one of them. At present, the main Internet users in my country are young people, and online language violence brings extremely serious psychological problems to young students. In order to understand the current mental health of young students and the impact of online language violence on them, this article investigates the students in the city's no. 1 middle school, filters the data through decision tree analysis, and judges online language through the psychological symptoms self-rating scale. The mental health symptom self-rating scale has the characteristics of large capacity, abundant symptoms, and more accurate description of the subject's conscious symptoms. It contains a wide range of psychiatric symptoms, from feelings, emotions, thinking, consciousness, and behavior to life habits, interpersonal relationships, eating, and sleeping, and it uses 10 factors to reflect the psychological symptoms in 10 aspects. It has good distinguishing ability for people with psychological symptoms (that is, they may be on the edge of psychological disorder or mental disorder). The chi-square statistical method is used to analyze the basic characteristics of different youth groups of verbal violence. For the research content, the school surveys all schools and adopts questionnaire surveys and case studies to analyze the factors that influence youths' attribution of online violence behaviors and make recommendations. The impact of violence on young students will be analyzed later through psychological intervention. The results of the study found that online language violence caused serious harm to young people's psychology and caused students' depression, anxiety, and other mental illnesses. Active psychological interventions can effectively alleviate students' mental health. The improvement of students' mental health is the most obvious. The score improved by nearly 10%.

## 1. Introduction

Young students in adolescence have extremely significant mental health problems. Young students are in a period of transition from childishness to maturity. This period is not only the key period of their physical and mental development, but also the most unstable period in their life. Their physiology tends to mature, but it fails to keep up with the pace of physiological development, which is very unbalanced. In addition, the inner world of young students is rich and colorful, but they are not easy to reveal. They have strong autonomy in psychology and behavior. They are sensitive, special, and active beings in social groups. Due to the lack of mature judgment for various external stimuli and the influence of various social undesirable phenomena, young people in development are increasingly exposed to their negative effects while enjoying the rich spiritual feast brought by the Internet. As a result, obsessions with online games, online chats, and even pornographic networks also happen from time to time. The constant occurrence of online immoral behaviors, especially online violence, has changed their original values and world outlook, giving them wrong guidance, and even induced some young people to become accomplices of online violence, and this also hinders them. The interests of society and others hinder the construction of socialist morality and spiritual civilization.

Social media has become a way for people to obtain information, and behaviors such as watching news, comments, and posting have also become a habit for people to express their feelings or thoughts [1]. But when people express their feelings or thoughts, there will be some “irrational” negative problems like language violence. Its appearance not only pollutes the virtual social environment, but also has an impact on people's lives and even causes a certain degree of damage to the human body or physiology. Especially, the “human keyboard” that has appeared in the virtual world in the past two years lead to problems such as “racism, sexism, general sympathy, false expressions, and moral kidnapping.” Thus, the Internet language violence is especially harmful to young students.

Experts at home and abroad have conducted many studies on the methods of mental health intervention for online language violence agents. Revita et al. discussed polite forms in the language of angry people. The data are collected by taking notes, recordings, and conducting interviews. Aiming at the concept of female verbal violence, a descriptive analysis of the survey results was carried out, and several tables were added to present some data [2]. Sari described verbal violence and expressive speech acts in the form of instructions in Kiko cartoon. The collected data were analyzed based on verbal violence in the form of command and expressive speech acts, grouped according to indicative and expressive speech acts [3]. Karni-Vizer and Salzer counted the oral and written language violence experienced by some people. 82% of participants reported at least one type of verbal violence in their lifetime, and 66% of participants reported incidents in the past year. It has a potentially destructive impact on mental health, well-being, and sense of security [4]. Hamzaoglu and Türk's statistics on the mechanical energy of language violence in the workplace showed that a total of 36.7% of the participants reported that they had experienced physical violence, and 88.8% of the participants reported that they had suffered at least one verbal abuse during their working life. Regulations on effective communication training, changing workplace conditions, and effective implementation of violence prevention procedures may help reduce the incidence of verbal abuse and physical violence [5]. Spijkerman et al. conducted 15 randomized controlled trials. The random effects model was used to calculate the effect size between the before and after groups, and the quality of each included trial was rated. Research results indicate that online MBI may help improve mental health outcomes [6]. Rice et al. used the adjusted risk of bias tool to assess the quality of the research; the quality of the evidence is rated according to the GRADE (Recommended Assessment, Development, and Evaluation Grading) standard. The most common mental health conditions are depression (19% (95% CI, 14%–25%)) and binge eating disorder (17% (95% CI, 13%–21%)) [7]. The purpose of Al-Zayyat and Al-Gamal's study is to determine the degree of stress perceived by undergraduate nursing students in the clinical practice of the PMHN course, the types of stressors, and coping strategies. The results of the study showed that the highest types of stressors reported during the two data collection periods were patient care, stress related to teachers and nursing staff, and stress from tasks and workload [8]. These studies provide a certain reference for this article, but due to the lack of rigorous experimental methods, the experimental results are difficult to reproduce, making the experimental results unconvincing.

This article is mainly aimed at the problem of language violence on the Internet, from a micro perspective to study the causes and diffusion process of Internet language violence. Research on the impact of online language violence was on the mental health of young students and intervention strategies, specifically using empathy theory, behavioral alienation theory, and stereotype theory to study the issue of language violence in social media comments. In recent years, the use of data mining technology to explore the mental health of college students and the mode of psychological crisis intervention has become a hot spot for scholars at home and abroad. Data mining technology was used to dig out the relationship between the various factors that cause students' psychological problems from the survey data and to determine the main factors that affect students' psychological problems, etc. The decision tree algorithm is used to analyze the mental health of students. The algorithm is not urgent, the principle is easier to understand, the calculation is not very large, the speed is fast, and the generated rules are easily understandable (suitable for psychological educators to understand decision-making). And because the characteristics of students are relatively fixed, real-time classification is not required, and the amount of calculation can be ignored, so the decision tree algorithm is more suitable for students' mental health analysis. This article not only enriches people's research results on online language violence, but also deepens people's understanding of online language violence. The generation of youth online violence has its profound family and social background. Through the research on the attribution methods of the results of online violence, we can provide effective attribution training guidance for future family and school moral education, namely, finding, from the results, the mechanism of influence on the occurrence of cyber violent behaviors plays a preventive role at the source, helps young people to obtain the correct attribution method, enhances the awareness of moral responsibility, and makes them dare to face reality and assume responsibility, which can not only effectively prevent the occurrence of unethical behaviors but can also improve the moral consciousness of young people and promote the development of moral behavior.

## 2. The Impact of Mental Health and Intervention Countermeasures

### 2.1. Classification of Online Language Violence

Regarding the types of online language violence, this article divides it into three categories according to the degree, characteristics, and meaning of language violence, divided by the form of language violence, by the direction of the incident, and by the gender of the user.

Internet language has developed rapidly because of the popularity of the Internet and spread rapidly because of the popularity of Internet communication. At the same time, Internet language can cause all aspects of traditional language in such a short period of time. The impact of this has aroused the attention of the whole society. In recent years, there have been a lot of articles on Internet language, and articles on the influence of Internet and online communication on young people are also emerging. However, few articles have studied the influence of Internet language on young people. This article can make the overall content more focused.

According to its form, cyber violence can be divided into pure text language violence, pure image language violence, pure expression language violence, text plus picture language violence, text plus emoticon language violence, and picture plus emoticon language violence [9]. In general, this article divides the verbal violence in social media comments into three types, namely text and language violence, image language violence, and emoji violence. Among them, language violence in the text refers specifically to the violence in the text language [10]. It does not only include pure verbal violence but may include image language violence, image and text-based language violence, and also image-type language violence plus emoticons. Violence in graphic language includes violence in language and expressions plus language text.

Language violence was in social contradictions. It comes from the projection of real life on virtual social platforms; that is, the language of cyberbullying reflects the psychological pressure people have accumulated in real life, such as anger, disgust, hatred, and resentment. Since these pressures cannot be vented in real life, they can only vent on the virtual online world [11].

Cyberspace is close to Kant's formlessness, and it is a virtual space that is close to infinity. Writing on Weibo on the Internet and expressing one's opinions on forums and posts are a very simple matter. In addition, the censorship system is very loose, which makes expression easier [12, 13]. Network information is gathered and updated at a rapid rate, and various opinions will spread in a snowball way. It is the openness of the Internet that makes it easier to spread language violence. The basic composition of language violence is shown in Figure 1.

In addition, the anonymity of the Internet also adds “tiger wings” to the “verbal violence” of enterprises. On the one hand, anonymous communication protects the rights of netizens to freedom of speech, but on the other hand, it also weakens netizens' sense of moral responsibility and binding force [14, 15]. In the network communication environment, the weakness of human nature is at a glance, but under the cover of anonymity, netizens do not have the moral cultivation and professional ethics of traditional media communicators, and their behavior is not restricted by political systems and laws at all [16, 17].

The Internet is a bottomless pit, and there are no rules for its entry and exit. In network communication, one party sends out a message, and thousands of other parties respond unanimously. This kind of interaction makes the network communication extremely ambitious. In the process of this dissemination, there is no “gatekeeper” to screen and supervise the information, which causes the information to enter indiscriminately and has a negative impact on the dissemination environment [18]. Although there is a “microblogging secretary” on Weibo as a supervisor, it does not play a major role in purifying the entire Weibo communication environment.

Secondly, there are hidden dangers in network security technology. In Internet communication, netizens can use some technical means, such as human flesh search, to dig out the true identity of netizens, expose others' privacy through online channels, and create conditions for language violence and personal attacks [19, 20]. Third, with the continuous development of human communication, the current mass media has entered the era of network communication, and its influence surpasses any previous media forms. According to CNNIC statistics, Chinese Internet users have reached 668 million. Network communication covers a wide range of people, more than any previous medium [21]. Network language originates from network communication, and the research of network communication involves many disciplines such as philosophy, sociology, communication, informatics, psychology, and pedagogy. Due to the increasing popularity of online communication, online language spreads and develops among netizens with an unstoppable momentum. Over the past decade or so, online languages have changed from little known to popular to language fashion. From activities in virtual spaces on the Internet, the community of netizens with the characteristics of independence, openness, tolerance, diversity, and innovation has gradually entered the real society and has gradually created and formed network language with its own characteristics.

Many websites deliberately fan the flames in order to cater to the market and pursue a sensational effect when hot issues break out, making things more and more influential. In online language violence, whether it is a scolding war or a face-slapped incident [22], website operators see these violent language conflicts but do not stop them and let them develop. The purpose is to increase visibility, bring in more traffic, and increase website revenue. Language is the main medium through which we implement education, and education in turn can regulate and manage language. At the same time, the culture and expression carried by language are closely related to the progress of human civilization, people's thinking, and the construction of the world outlook. The article uses a decision tree algorithm to discriminate and analyze online language violence, so the overall content of the article is very logical.

The “helpers of abusers” of language violence are netizens in the Internet age, and their behavior directly leads to and deepens the language violence of competing companies [23]. In addition, on the Internet, the quality of netizens is uneven. According to the statistics report on the development of the Internet, middle school and high school netizens are the main body and core of the entire netizens. The number of netizens with elementary school and below is gradually increasing, and Chinese netizens are gradually turning to be low educated. These netizens of different age levels, different educational levels, and different occupations must have different qualities and therefore have different behaviors on the Internet. Due to the intermediary nature of language contact and language, young people are impacted by online language at the stage where the language model is not solidified, so it is easy to change their language views and language forms. Young people are affected by the Internet culture before their outlook on life and values are clearly defined, and they will easily have an impact on the youth who are in the process of forming their outlook on life and the world. So this comes from the evolving network culture.

### 2.2. Information Processing Methods

With the continuous progress and development of information technology, the amount of all kinds of effective and useful data continues to increase sharply. There is a wealth of knowledge in these data, and the most urgent task at present is to find valuable information from the massive data and transform this information into organized knowledge. Different data mining methods need to be used for different types of data. Decision tree algorithm is an important method of classification and a typical data mining technique [24]. Decision tree algorithm, as a simple, efficient, and highly explanatory model, is widely used in the field of data analysis. The realization principle of the decision tree is shown in Figure 2.

In the decision tree algorithm, the optimal split attribute feature can well reflect the classification of tuples, and the classification requires less relevant information. For the algorithm itself, it reduces a certain amount of work and improves efficiency. Below is the expectation of set *D*.

(1) $$\begin{array}{c} \text{Info}\left(D\right)=-\overset{m}{\underset{i=1}{\sum }}p_{i}\log\;2\left(p_{i}\right). \end{array}$$

Here, *p*_*i*_ represents the probability that the sample in the set *D* belongs to the class *C*_*i*_, and it is calculated by using *C*_*i*_ for related evaluation.

In the decision tree classification process, according to the attribute feature A, to classify the sample set, perform downward branching, and then get the required expected information:

(2) $$\begin{array}{c} {\text{Info}}_{A}\left(D\right)=\overset{v}{\underset{j=1}{\sum }}\begin{array}{c} Dj\\ D \end{array}*\text{Info}\left(D_{j}\right). \end{array}$$

The difference between the old information demand and the new demand represents information gain, and the specific expression is as follows:

(3) $$\begin{array}{c} \text{Gain}\left(A\right)=\text{Info}\left(D\right)-{\text{Info}}_{A}\left(D\right). \end{array}$$

The algorithm uses the information gain ratio index to select the optimal split point. The gain information ratio can avoid dependence on attribute features with a large number of values when selecting the optimal attribute feature. It can maximize the classification performance of the decision tree. The split information is defined as follows:

(4) $$\begin{array}{c} \text{Split }{\text{Info}}_{A}\left(D\right)=-\overset{v}{\underset{j=1}{\sum }}\begin{array}{c} D_{j}\\ D \end{array}*-\;\log_{2}\left(\begin{array}{c} D_{j}\\ D \end{array}\right). \end{array}$$

Calculate the information gain ratio, and find the optimal splitting attribute feature, as shown in the following formula:

(5) $$\begin{array}{c} \text{Gain Ratio}\left(A\right)=\begin{array}{c} \text{Gain}\left(A\right)\\ \text{Split }{\text{Info}}_{A}\left(D\right) \end{array}. \end{array}$$

This paper uses independent sample verification method to select the best subtree in the subtree sequence {*T*_0_, *T*_1_, *T*_2_,…, *T*_*n*_}. Split the large-scale training set *C* into two independent sample sets *C*_1_ and *C*_2_, where the number of instances of *C*_2_ is *n*. Let *n*_*j*_ represent the number of instances of category *j* in *C*_2_; the predicted probability can be obtained from

(6) $$\begin{array}{c} P\left(i|j\right)=\frac{n_{ij}^{2}}{n_{j}^{2}}. \end{array}$$

The misjudgment cost of its category:

(7) $$\begin{array}{c} R\left(j\right)=\sum_{i}c\left(i|j\right)P\left(i|j\right). \end{array}$$

Among them, *c*(*i*|*j*) is the cost value of the sample of category *j* that is judged to be category *i*. The misjudgment cost of its subtree *T* is

(8) $$\begin{array}{c} R\left(T\right)=\sum_{i}R\left(j\right)P\left(j\right). \end{array}$$

Suppose that the parallel shared decision tree constructed according to the data set pair (*D*_1_, *D*_2_) is *T*, that is,

(9) $$\begin{array}{c} \text{Acc }D_{i}\left(T\right)=1-\begin{array}{c} 1\\ \text{mum}D_{i} \end{array}\overset{n}{\underset{j=1}{\sum }}W_{j}. \end{array}$$

Among them, *D*_*i*_ represents the data set, *W*_*j*_ represents the number of tuples misclassified by *D*_*i*_ on node *j*, and mum*D*_*i*_ is the total number of *D*_*i*_ tuples. Given a node V on the parallel shared decision tree *T*, the class distribution vector *D*_*i*_(*i*=1,2) of the data set at node V is

(10) $$\begin{array}{c} CDVi\left(V\right)=\overset{n}{\underset{j=1}{\sum }}C\;DV_{ij}\left(v\right). \end{array}$$

(11) $$\begin{array}{c} CDV_{ij}\left(V\right)=\left(Cnt_{ij}\left(C_{1},V\right),Cnt_{ij}\left(C_{2},V\right),\ldots ,Cnt_{ij}\left(C_{k},V\right)\right). \end{array}$$

Here, *n* is the number of computing nodes in the cluster, *D*_*i*_ represents the data set, and *C*  *DV*_*ij*_(*C*_*k*_, *V*) is the number of tuples *D*_*i*_ stored in computing node *j*.

Simplify the calculation by taking the absolute value method, and get

(12) $$\begin{array}{c} M_{n}=\sum_{m=-\infty }^{\infty }\left|x\left(m\right)\right|w\left(m-n\right)=\sum_{m=n}^{n+N-1}\left|x_{w}\left(m\right)\right|. \end{array}$$

The number of signal zero-crossings refers to the number of times the signal amplitude value changes from positive to negative or from negative to positive. The short-term zero-crossing rate refers to the number of times the signal passes the zero value in each frame in a short period of time, defined as

(13) $$\begin{array}{c} Zn=\frac{1}{2}\overset{\infty }{\underset{m=-\infty }{\sum }}\left|\mathrm{sgn}\left[x\left(m\right)\right]-\mathrm{sgn}\left[x\left(m-1\right)\right]\right|w\left(n-m\right), \end{array}$$

where sgn represents a sign function, as shown in the following formula. When sgn is nonnegative, the function value is less than 1. When *n* is less than 0, it is a window function.

(14) $$\begin{array}{c} \mathrm{sgn}\left[n\right]=\left\{\begin{array}{c} 1\begin{array}{c} \;n\geq 0 \end{array}\\ -1\;\begin{array}{c} n\leq 0 \end{array} \end{array}\right.. \end{array}$$

Assuming that the input of the system training data is *X* and the expected output value is *Y*, then the general input formula of each neuron in the hidden layer is

(15) $$\begin{array}{c} H_{j}=\overset{n}{\underset{i=1}{\sum }}\varphi_{ij}x_{i}. \end{array}$$

Through the study of Internet language, to analyze its impact on young people, it is recommended to guide the use of Internet language by young people through educational means, so as to promote the healthy development of youth culture. This part of the article uses a decision tree method. Generally speaking, changes in parameters have a certain impact on the article results, but this part of the article has little effect on this parameter, so Sigmoidal can ignore the impact. In order to simplify the calculation, the value in Sigmoidal *φ* is usually set to 1; then, the output results of each hidden node can be obtained:

(16) $$\begin{array}{c} {\text{net}}_{j}=f\left(H_{j}\right)\;j=1,2,...,l. \end{array}$$

The input of each output node is

(17) $$\begin{array}{c} O_{k}=\overset{1}{\underset{j=1}{\sum }}H_{j}w_{jk},\;k=1,2,...,m. \end{array}$$

Suppose we expect the value of the *i*-th output neuron to be *d*_*i*_, then the prediction error of the *i*-th neuron is *e*_*i*_=*d*_*i*_ − *y*_*i*_, and then the error function of the output layer is

(18) $$\begin{array}{c} E=\frac{1}{2}\sum_{i}e_{i}^{2}=\frac{1}{2}{\left(d_{i}-y_{i}\right)}^{2}. \end{array}$$

Therefore, the error data transfer equation between the input layer and the hidden layer is

(19) $$\begin{array}{c} \Delta \varphi_{ij}=-\eta \frac{\partial E}{\partial \varphi_{ij}},\;i=1,2,...,n. \end{array}$$

Because of the sigmoid function *f*′(*x*)=1*f*(*x*)(1 − *f*(*x*)), the result is

(20) $$\begin{array}{c} \Delta w_{jk}=-\eta \left(d_{i}-y_{i}\right)y_{i}\left(1-y_{i}\right){\text{net}}_{j}. \end{array}$$

The limitations of objective technology and the desire to save input time and Internet fees subjectively are the fundamental reasons for the emergence of online language. Saving input time and surfing expenses is the direct demand of young netizens and the motivation of net language. The material foundation of the net provides the possibility and restriction condition of the net language method which is the technical condition. The mathematical model constructed by the algorithm has very rigorous characteristics and at the same time has good learning ability, good fault tolerance, and good generalization. The data processing flow is shown in Figure 3.

### 2.3. Evaluation and Intervention of Psychological Symptoms

The self-reference index for physical and psychological symptoms (SCL-90) is related to all dimensions of MSQA. The symptom self-rating scale was created by Derogatis in 1975 [25]. The scale has a total of 90 items, and each item uses a score of 1–5. A score scale of 1 indicates that there is no such problem; a score of 2 indicates very mild problem; that is, there are symptoms but no actual effect or low effect; 3 points indicate moderate symptoms: there is a certain effect; 4 points indicate that the symptoms are severe and have a certain effect; 5 points indicate that the symptoms are very severe. Young students are generally 15–18 years old, and they are in adolescence. It is a critical period of physical and psychological development, and it is also a stormy stage, which is prone to psychological conflict and psychological confusion. Some previous studies have shown that there are many factors influencing the development of mental health of secondary vocational students, including family environment, school education, social culture, genetics, and individual factors, [26]. Network language and network culture are a kind of cultural phenomenon associated with network technology. The young netizen community has the characteristics of independence, openness, tolerance, diversity, and innovation. They despise tradition, have a strong antitraditional consciousness, and advocate innovation. Ideologically, it is completely free from the constraints of traditional language grammar and semantic norms and standards. In reality, the in-depth English education has given contemporary young people more corpus resources than in the past, so it can create a convenient network application language form.

At present, the current situation of young people's learning mental health is not optimistic. Family, school, social, and individual's own factors will affect their mental health development. They need to receive more positive attention. Therefore, the secondary vocational students are the research objects: their mental health status and influencing factors, giving them correct guidance and education and improving their mental health level, in order to provide a basis for the school's mental health education [27].

Generally speaking, offering mental health courses or psychological counseling can play a role.

First, teachers of mental health courses teach college students the basic theories and basic knowledge of psychology and mental health. This includes not only the concept of mental health, the standards of mental health, but also the goals of mental health, the content of mental health, and so on.

Second, teachers of mental health courses teach college students the skills and methods for overcoming psychological barriers and adjusting psychological problems. This includes establishing what kind of correct inner thoughts and what kind of active and healthy behaviors.

Third, teachers who combine the teaching content of mental health education provide collective counseling for the mental health problems that are common to the whole class. For example, with the help of beautiful music, students can recite poems and express their inspiration for art to judge their inner psychological emotions and state.

Fourth, teachers who combine the teaching activities of mental health education conduct one-on-one individual consultations on the individual psychological problems and obstacles of college students. For example, every student is asked to write down the troubles and confusions in his life and study and then hand them to the teacher for individual counseling.

All in all, in the process of mental health education courses, psychology teachers explain mental health knowledge and skills and combine the content of mental health teaching, interspersed with various psychological counseling and mental counseling to act on the mental health of college students and make them psychologically healthier. The level of health tends to be improved.

In addition to rich information, the most direct benefit that the Internet brings to people is the civilianization of the right to speak. Some people call this era the era of language riots. The Internet provides everyone with a stage for self-expression, and performance gives everyone a unique space to express their individuality and release themselves. When real people communicate in the virtual world, online language becomes their catharsis tool in this community; in real communication, it is borrowed as a convenient and casual communication medium for them.

Everyone has three basic needs in the process of interpersonal communication: tolerance, control, and emotional needs. These three needs determine the behavior of individuals in interpersonal communication and how to interpret and predict the behavior of others. The need for tolerance refers to the individual's need to be accepted by the team, communicate with others, and establish good relationships with others. In the process of individual development, if the need for tolerance is not met, they will behave at a distance from others and the group, forming low social behavior; if the need for tolerance is met, satisfied people will very much want to contact people to form super social behaviors [28]. Sovereignty needs refer to the needs of individuals who want to dominate or be dominated by others and check and balance each other in the distribution of power. If an individual is in a democratic and free environment when he/she is young, he/she will be very aware of their status and power. When they get along with others, they will be in a state of balance between having control and being controlled. When a person is young in an authoritarian or simple environment, their behavior will tend to be authoritarian or submissive. Authoritarians demand that others obey their orders and want complete control. The obedient person has no opinion of their own and is always willing to act as a supporting role. Online language violence originates from online communication. With the popularization of the Internet, the use of Internet instant messaging and chatting has become one of the main functions of Internet use, and Internet interpersonal communication has increasingly become a part of modern life. Since its inception, it has been rapidly popularized and developed mainly among young netizens. Under the current development situation, it has become a focus of social attention due to the scale of the population.

## 3. Intervention Experiments and Results

### 3.1. Learning Mental Health Status

We take the city's no. 1 middle school as an example to conduct surveys and statistics on students and teachers. The results are shown in Table 1.

It can be seen that the detection rate of seniors and boys is higher. The two dimensions of emotional problems and social adjustment difficulties are particularly obvious in mental subhealth. The number of positive entries in these two dimensions is shown in Table 2.

Since we want to compare online language violence, we first classify the current population on the Internet and analyze the educational structure of netizens in the past two years according to their educational background. The results are shown in Figure 4.

As can be seen from the figure, the statistical results of the past two years show that the current netizens are relatively small, mainly concentrated in junior high and high school students. This part of the population accounts for about 70% of the total. Therefore, the sample we chose is also the city's no. 1 middle school.

We investigated whether the experimenters suffered from online language, and the results are shown in Table 3.

The basic characteristics of the three groups of youths suffering from language violence were analyzed using chi-square statistics, and the results are shown in Table 4.

The results showed that among the adolescents who did not suffer from language violence, 65 were males, accounting for 39.6%, and 101 were females, accounting for 60.4%. Among the adolescents who rarely suffered from language violence, 53 were males, accounting for 52.8%, and 47 were females, accounting for 47.2%. Among the teenagers who frequently suffered from language violence, 204 were males, accounting for 82.7%, and 41 were females, accounting for 17.3%. The difference in gender is statistically significant (*P* < 0.001). There are more male adolescents suffering from language violence.

As for the impact of language violence on young people's learning psychology, we conducted relevant surveys and statistics, and the results are shown in Figure 5.

It can be seen that in the case of online language violence, 392 (76.4%) with emotional problems are normal, 93 (18.1%) are average, and 28 (5.5%) are abnormal. 400 (78.0%) with character problems were normal, 72 (14.0%) were average, and 41 (8.0%) were abnormal. The scores of hyperactive attention deficit problem were 400 (78.0%) normal, 57 (11.1%) average, and 56 (10.9%) abnormal. 417 (81.3%) with same-age communication problems were normal, 75 (14.6%) were average, and 21 (4.1%) were abnormal. 393 (76.6%) with social behavior problems were normal, 74 (14.4%) were average, and 46 (9%) were abnormal. The total difficulty of 345 (67.3%) was normal, of 120 (23.4%) was average, and of 48 (9.4%) was abnormal.

### 3.2. Intervention Comparison

We surveyed students who suffered language violence and compared their mental health scores before and after other interventions. The results are shown in Figure 6.

It can be seen from Figure 6 that there are very significant differences in the physical subhealth scores of the experimental group before and after the intervention, except for the sleep problem factor. This shows that after Internet language violence, through intervention methods, students' subhealth conditions can be effectively reduced. In order to select effective data, we conducted multiple tutoring with relevant students. After that, we calculated the data and took the average of the data. The result is shown in Figure 7.

It can be seen from the average value that the scores before and after the intervention have changed to a certain extent. The scores of the self-rating symptom scale of the experimental group have significant differences in interpersonal relationship sensitivity and anxiety before and after the intervention, and there are very significant differences in the total scores. After a period of time, some students who did not undergo intervention were evaluated again. The mental subhealth of the control group was equally scored before and after the intervention. The standard deviation is shown in Figure 8.

It can be seen that the average score of the psychological counseling intervention is higher than that of the pretest, and the difference has reached an extremely significant level. Among them, the scores of learning and social interaction are significantly higher than those before the intervention, and there are extremely significant differences. We conducted a statistical analysis of the physical subhealth before and after the intervention, and the results are shown in Figure 9.

The mean and standard deviation of the symptom self-rating scale before and after intervention in the control group are shown in Figure 10.

It can be seen from the figure that the symptoms of online language violence have changed before and after the intervention. Among them, the mental condition of the students has improved the most, with a score improvement of nearly 10%, and other symptoms have also improved to varying degrees. The mean and standard deviation of the symptom self-rating scale after the intervention in the control group were not lower than that before the intervention, and there was no significant difference.

## 4. Discussion

### 4.1. Students' Mental Health

In social media, virtual environments amplify personal dissatisfaction, and information closely related to individuals can easily lead to verbal violence. The degree of personal complaint mainly depends on two factors: on the one hand, the influence of emotional tendency on personal language comments, and, on the other hand, the influence of selfishness on personal language comments.

Gender, grade, peer structure, and family residence do not affect mental subhealth. In this study, the overall mental subhealth status of high school students did not find such a difference. The chi-square test found that the values of the mental subhealth status of high school students and their gender, grade, peer structure, and family residence were 0.416, 0.268, 0.706, and 0.688, respectively, which were all greater than 0.05, indicating that there was no significant difference between them. This shows that after high school students are subjected to online language violence, mental subhealth problems are more common, and there is no difference in gender, grade, peer structure, or family residence. The reason for this phenomenon may be the development of the current era and society, as well as the fierce competition for talents. The concern of schools and families for high school students is currently mainly focused on their academic performance. The heavy academic work makes the students get very bored. Life is more depressing, making them unable to find a suitable space and time to relax. At present, if schools, families, and society do not pay more attention to physical and psychological health development of student's personality, abilities, and other aspects, then academic pressure may cause them to be overwhelmed.

### 4.2. Suggestions for Improvement

The media plays a vital role in disseminating information, especially in virtual social networking, where every word and deed of the media can guide public opinion. Therefore, the basic theoretical knowledge of the media and the knowledge of media operators need to be improved. A skilled media operator must not only have a solid basic theoretical knowledge and the ability to reason about others but also be able to display various information, suspicions, knowledge, and crises on social media. To enjoy the media and media resources better, correctly and faster, so as to improve oneself and create a beautiful virtual social environment, the media should also enhance the guiding role of public opinion.

Netizen users are the basis for the survival of social media, because ordinary netizen users are the most used and largest social media group. It claims that Internet users use civilized language. As the saying goes, “one pass ten, ten pass a hundred”; thus, the behavior of people under the group psychology is blind, and it is also one of the reasons for the emergence and proliferation of language violence on social media. The civilization of virtual social space is inseparable from ordinary users of the Internet. In addition, it is necessary to strengthen the education of virtual society laws and regulations for ordinary netizens, to address the problems of virtual social platforms, formulate relevant laws and regulations, encourage ordinary users to learn and use social media, and be civil and healthy users.

The experimental results of this article showed that after the psychological intervention of the students, the survey was conducted again, and it was found that the number of mentally subhealthy people in the experimental group was reduced to 15, accounting for 37.5% of the total. Although the average score of each factor decreased, there were still more people in the control group who were mentally subhealthy. The number of healthy people is still 12, but most of the factor scores are higher than two months ago. According to the results, there are significant differences in the average scores and standard deviations of the factors in the experimental group before and after the intervention. There are only significant differences in the standard deviation of mental subhealth before and after the intervention in the control group, but there is no significant difference in the average scores and standard deviations between the experimental group and the control group after the intervention, which shows that the intervention effect of group counseling on mental subhealth is not obvious, and it has not played a significant positive effect. The significant difference between the pretest and posttest results may be due to time, an irrelevant variable, which played a role in the middle, or it may be due to the fact that group counseling, an intervention measure that does not have a positive impact on mental subhealth, should be combined with other methods.

From the data after this group counseling intervention, it can be found that the intervention effect of short-term group counseling on mental subhealth is limited. This may be because psychological problems themselves are a complex, internal, and long-term evolutionary process. The improvement of psychological problems requires the coordination and participation of multiple factors and methods, and group counseling alone cannot achieve overall improvement of the role of mental subhealth. If we want to transform the mental subhealth state into a mental health state, we need to use a variety of methods to make adjustments in all aspects of life, pay attention to cultivating good psychological qualities, strengthen psychological stress resistance, and form a positive and optimistic attitude.

## 5. Conclusions

On the Internet, virtual environments reflect social contradictions, and information related to social contradictions can easily lead to language violence. In a virtual society, social conflicts mainly stem from differences in regional culture and changes in social roles. The former caused linguistic conflicts among people, and the latter caused verbal violence among them. In short, people have aggravated social contradictions due to differences in regional culture and changes in social roles. The relationship between virtual social interaction and gender was “identification.” In social media, the virtual environment deepens the “identity” of gender. In terms of verbal violence, women are stronger than men. When young students communicate online, they should communicate in a civilized manner to avoid becoming victims of online language violence. Of course, the research in this article also has some shortcomings. The subject samples of this study are relatively small. Due to time, environment, and capacity constraints, the object of this study is only the city's no. 1 middle school, and the sample types are insufficient, making it difficult. Involving all kinds of young students, there are certain differences in experimental results. In future research, it is necessary to strengthen the data sample and strive to obtain more rigorous results.

## Figures and Tables

**Figure 1:** Composition of language violence.

**Figure 2:** Implementation schematic.

**Figure 3:** Data preprocessing process.

**Figure 4:** Changes in the structure of netizens.

**Figure 5:** Mental health impact.

**Figure 6:** Scores before and after psychological intervention.

**Figure 7:** The scores of the experimental group before and after intervention.

**Figure 8:** Comparison before and after mental subhealth intervention.

**Figure 9:** Physical subhealth changes.

**Figure 10:** Control group before and after intervention.

**Table 1:** Survey results.

Classification		Mental health		Total	Detection rate (%)
		Yes	No		
Grade	High school	162	34	196	17.6
	Sophomore	125	50	175	32.1
	Senior three	106	59	165	35.9

Gender	Male	152	65	217	29.7
	Female	236	86	322	26.7

Peer structure	Only child	159	64	223	28.8
	More than one child	229	86	315	27.3

Home residence	The city	244	92	336	27.4
	Rural area	144	58	202	28.8

Teacher	Young teacher	58	12	70	17.1
	Middle-aged teacher	62	10	72	13.9
	Senior teacher	35	20	55	36.4

**Table 2:** Number of mental subhealth items.

Dimension	Factor	Number of people	Proportion (%)
Emotional problems	1 anxiety, depression	148	39.6
	8, 9 horror	58	15.6
	12 suicide	17	4.7

Social adaptation	2 learning difficulties	167	44.7
	7 social discomfort	86	23.1

**Table 3:** Online language violence.

Classification	Number of cases (*n*)	Percentage
Not subjected to violence	165	32.2
Rarely suffered from violence	101	19.8
Often subjected to violence	244	48
Total	510	100

**Table 4:** Language violence experienced by young students.

Classification	Not subjected to violence		Rarely suffered from violence		Often subjected to violence		*χ* ^2^	*P*
	Number of cases (*n*)	Percentage	Number of cases (*n*)	Percentage	Number of cases (*n*)	Percentage		
Gender								
Male	65	39.6	53	52.8	204	82.7	84.2	0.001
Female	101	60.4	47	47.2	41	17.3		
Age								
12-13	74	45.2	43	42.9	104	42.7	0.79	0.928
14-15	81	49.2	52	50.8	121	49.6		
16-17	11	5.6	7	6.3	20	7.7		

## Data Availability

The data that support the findings of this study are available from the corresponding author upon reasonable request.

## References

[1] Li X., Jianmin H., Hou B., Zhang P. (2018). Exploring the innovation modes and evolution of the cloud-based service using the activity theory on the basis of big data. *Cluster Computing*.

[2] Revita I., Triclarise R., Anggraini N., Gunawan F. (2020). Politeness IN domestic verbal violence against women IN Indonesia. *Aksara*.

[3] Sari I. A. R. (2020). Kekerasan verbal dalam film kartun KIKO(verbal violence IN the KIKO cartoon film). *Jurnal Bahasa, Sastra Dan Pembelajarannya*.

[4] Karni-Vizer N., Salzer M. S. (2016). Verbal violence experiences of adults with serious mental illnesses. *Psychiatric Rehabilitation Journal*.

[5] Hamzaoglu N., Türk B. (2019). Prevalence of physical and verbal violence against health care workers in Turkey. *International Journal of Health Services*.

[6] Spijkerman M. P. J., Pots W. T. M., Bohlmeijer E. T. (2016). Effectiveness of online mindfulness-based interventions in improving mental health: a review and meta-analysis of randomised controlled trials. *Clinical Psychology Review*.

[7] Rice S. M., Purcell R., De Silva S., Mawren D., McGorry P. D., Parker A. G. (2016). The mental health of elite athletes: a narrative systematic review. *Sports Medicine*.

[8] Al-Zayyat A. S., Al-Gamal E. (2016). Perceived stress and coping strategies among Jordanian nursing students during clinical practice in psychiatric/mental health courses. *International Journal of Mental Health Nursing*.

[9] Dos S., Carlos B. J., Cecilio H. (2017). Ayahuasca: what mental health professionals need to know. *Arch. clin. psychiatry*.

[10] Cardoso G., Xavier M., Vilagut G. (2017). Days out of role due to common physical and mental conditions in Portugal: results from the WHO World Mental Health Survey. *BJPsych Open*.

[11] Masykuroh Q. (2016). Physical and verbal violence IN Indonesian folktales retold IN children’S BOOKS. *Kajian Linguistik dan Sastra*.

[12] Park J.-C., Kwon H.-B. (2018). The effects of the employees self encouragement based on verbal violence in the workplace of hotel enterprise on anger express and turnover intention. *Korean Journal of Hospitality & Tourism*.

[13] Kim J.-K., Cho M.-S. (2019). The effects of verbal violence among hotel employees’ on job stress, job burnout, and job performance. *Journal of Tourism and Leisure Research*.

[14] Ryoo J. S.-C., Lee H.-J., Lee Y.-O. (2019). A study on the development of verbal violence and verbal defense curriculum for middle school students. *Korean Education Inquiry*.

[15] Khatwani G., Srivastava P. R. (2018). Impact of information technology on information search channel selection for consumers. *Journal of Organizational and End User Computing*.

[16] Kim M.-J., Lim C.-Y. (2017). Relationships between experiencing verbal violence and the emotional responses and coping behaviors of dental hygienists. *Journal of dental hygiene science*.

[17] Yu P., Zhou F., Zhang X., Qiu X., Kadoch M., Cheriet M. (2020). Deep learning-based resource allocation for 5G broadband TV service. *IEEE Transactions on Broadcasting*.

[18] Youn S., Cho T., Cho T., Yook P. (2016). Effects of casino employees-perceived verbal violence and a superior’s impersonal supervision on job satisfaction and turnover intention. *Journal of Tourism Management Research*.

[19] Yang Y., Li Z. (2017). Association between hypertension and emotional disorders: effect of psychological intervention. *Zhonghua xin xue guan bing za zhi [Chinese journal of cardiovascular diseases]*.

[20] Evans-Lacko S., Aguilar-Gaxiola S., Al-Hamzawi A. (2017). Socio-economic variations in the mental health treatment gap for people with anxiety, mood, and substance use disorders: results from the WHO World Mental Health (WMH)\\\\\\\\udsurveys. *Psychological Medicine*.

[21] Benotsch E. G., Zimmerman R. S., Cathers L. (2016). Use of the Internet to meet sexual partners, sexual risk behavior, and mental health in transgender adults. *Archives of Sexual Behavior*.

[22] Carson J., Cavagin J., Bunclark J. (2016). Effective communication in mental health nurses: did social support save the psychiatric nurse?. *NT Research*.

[23] Leslie S. (2016). Culture and mental health in the rainbow nation: transcultural psychiatry in a changing South Africa. *Transcultural Psychiatric Research Review*.

[24] Mohr D. C., Zhang M., Schueller S. M. (2017). Personal sensing: understanding mental health using ubiquitous sensors and machine learning. *Annual Review of Clinical Psychology*.

[25] Zivin K., Bohnert A. S. B., Mezuk B. (2016). Employment status of patients in the VA health system: implications for mental health services. *Psychiatric Services*.

[26] Zhang X., Zhang X., Chen X. (2017). Happiness in the air: how does a dirty sky affect mental health and subjective well-being?. *Journal of Environmental Economics and Management*.

[27] Mcleod G. F., Horwood L. J., Fergusson D. M. (2016). Adolescent depression, adult mental health and psychosocial outcomes at 30 and 35 years. *Psychological Medicine*.

[28] Harvey S. B., Modini M., Joyce S. (2017). Can work make you mentally ill? A systematic meta-review of work-related risk factors for common mental health problems. *Occupational and Environmental Medicine*.

